The article "Application of Care Bundles in Postanesthesia Recovery for Elderly Patients with Colorectal Cancer" was retracted in 2023. Reasons: unreliable results or conclusions; lack of ethics approval or compliance; concerns about the data; concerns about the peer review.

# Application of Care Bundles in Postanesthesia Recovery for Elderly Patients with Colorectal Cancer

**DOI:** 10.1155/2022/7669889

**Published:** 2022-06-21

**Authors:** Xiaoling Yu, Lichai Chen, Shuyi Chen, Weiming Qian, Lili Fang

**Affiliations:** ^1^Department of Nursing, Recovery Room, Department of Anesthesiology, The Second Affiliated Hospital Zhejiang University School of Medicine, Hangzhou 310009, China; ^2^Department of Nursing, Operation Room, Department of Anesthesiology, The Second Affiliated Hospital Zhejiang University School of Medicine, Hangzhou 310009, China; ^3^Department of Anesthesiology, The Second Affiliated Hospital Zhejiang University School of Medicine, Hangzhou 310009, China

## Abstract

**Objective:**

Based on the postanesthesia recovery procedure for elderly patients with colorectal cancer, a care bundle program was conducted to validate its effectiveness.

**Method:**

According to the characteristics of elderly patients with colorectal cancer, five measures including respiratory management, circulatory stability, pain assessment, body temperature monitoring, and internal environment stability were integrated into one bundle. Postanesthesia care unit (PACU) care bundle program for elderly patients was developed and used to improve recovery care. The monitoring data of the pre-PACB group given care bundles were collected and compared with the data of the post-PACB group who were given conventional recovery care.

**Result:**

222 patients in post-PACB group had shorter intubation time than 291 patients in pre-PACB group (37.7 ± 24.4 min vs. 42.1 ± 23.3 min, *P* < 0.05). The length of stay in PACU was longer in pre-PACB group (89.9 ± 33.5 min vs. 81.6 ± 31.1 min, *P* < 0.05). More adverse events were found in the post-PACB group than in the pre-PACB group (72.1% vs. 34.0%).

**Conclusion:**

After general anesthesia of patients with colorectal cancer, the application of the care bundles can improve the quality of recovery, shorten the intubation time and the length of stay in PACU, and reduce the complications caused by anesthesia.

## 1. Introduction

Colorectal cancer is the second leading cause of cancer-related mortality worldwide [1], and surgery is necessary for treatment. Advancement in technology leads to more elderly patients undergoing surgery year by year [2]. Compared with the young and middle-aged patients, it is more complicated and challenging to manage the elderly patients perioperatively due to the increased risk of anesthesia and surgery caused by the systemic diseases and the organ dysfunction [3]. Therefore, high-quality perioperative management is needed to accelerate their postoperative recovery. Anesthetic-related complications are likely to occur if we deal with it improperly. Respiratory complications, especially respiratory failure, followed by cardiovascular complications, were the most common adverse events in elderly patients with colorectal cancer during recovery, and these events were more frequent with advancing age [4]. Cardiac and pulmonary complications are also a main cause for many of these patients being sent to ICU after surgery [5]. Serious complications, a prolonged stay in PACU, and even an increased risk of death will occur in these older patients if they are not treated early or properly during recovery. There are many reports about the perioperative management of older patients [6]. These perioperative management programs include conducting a through preoperative assessment, developing a targeted care program based on the results of the assessment, and strengthening the management of the anesthesia process, postanesthesia, medication, and fluid. But few reports of caring measures in PACU for elderly patients were found.

Care bundles are a set of safe and effective care interventions provided by medical workers when patients are treated under unavoidable risks [7]. It was first proposed by the Institute for Healthcare Improvement (IHI) in 2001, with the aim of helping medical workers to provide patients with the best medical care services and achieve better treatment outcomes [8]. Nursing using care bundles is one of the best ways to translate the results of evidence-based research into clinical practice, thus helping to improve the quality of clinical nursing. In this study, a care bundle program was developed and implemented to guide how to provide medical care for the elderly patients with colorectal cancer who were sent to PACU under general anesthesia and offer intervention care, to improve the quality of resuscitation, shorten the length of stay in PACU, and reduce the risk of postoperative complications and chances of being sent to ICU.

## 2. Material and Methods

### 2.1. Study Design

This was a single-center retrospective study conducted at a tertiary hospital (the Second Affiliated Hospital, Zhejiang University). The study subjects were elderly patients undergoing colorectal cancer surgery between March 2020 and February 2021. Two periods were defined, based on the history of the postanesthetic care bundle (PACB): pre-PACB stage (March 2020-August 2020) and post-PACB stage (September 2020-February 2021). This study was approved by the ethics committee of the Second Affiliated Hospital of Zhejiang University (2021-0937). The categories of colorectal cancer surgery included laparoscopic, laparoscopic robot-assisted, and open resection for colorectal cancer. Data were collected from patients who met the following eligibility criteria. The inclusion criteria were (1) age 65 years or older, (2) a diagnosis of colorectal cancer, (3) treatment by colorectal cancer surgery under endotracheal general anesthesia, and (4) admission to postanesthesia care unit (PACU) postoperatively. The exclusion criteria were (1) presence of pulmonary infection, (2) presence of renal insufficiency, and (3) plan of recovery in the operating room or admission to intensive care unit (ICU) following surgery.

### 2.2. Caring Method Pre-PACB Stage

The patients in the pre-PACB group were treated with conventional recovery caring methods. After transferred to PACU, these patients were given assist control ventilation and synchronized intermittent mandatory ventilation, ECG monitoring, symptomatic treatment, and body temperature measurement. If body temperature is lower than 36°C, active warming was provided. Besides, after muscle strength was restored, the tracheal catheter was removed according to the doctor's advice. After extubation, the condition of the patients was continuously observed. If signs of respiratory depression or decrease in SPO_2_ were found, they were instructed to take deep breaths and cough properly. After they met the requirements to be transferred out of PACU, they would be sent to the ward after assessment by anesthesiologists. The nursing methods of pre-PACB group and post-PACB group are shown in Table 1.

### 2.3. Development and Implement of the PACB

#### 2.3.1. Development of the PACB

The PACB was developed from the evidence obtained from a few guidelines and expert consensus in the United States and China [9–15]. These bundled approaches include the following: (1) when patients should be extubated, (2) maintenance of circulatory homeostasis, (3) effective postoperative analgesia, (4) monitoring of body temperature, and (5) balance of internal environment. The above five key interventions are summarized to form a “bundle” of management program (Table 1) for postanesthesia recovery care.

#### 2.3.2. Implementation of the PACB

The PACB team consists of twelve PACU nurses and one anesthesiologist. The anesthesiologist is responsible for the evaluation of perioperative anesthesia and the management of multimodal analgesia. PACU nurses are responsible for the care of all patients and the recording of related monitoring data. Prior to implementation of the PACB, the head nurse gave the PACU nurses a train of three 30-minute courses on temperature monitoring, early extubation procedure, mechanical ventilation setting, assessment of respiratory function, clinical assessment of muscle strength recovery, monitoring of circulatory function, and pain assessment. We used the verbal rating scale (VRS) for pain assessment: grade 0: no pain; grade 1: mild pain. Although there is pain, it can be tolerated and can live normally. Sleep is not disturbed. Grade 2: moderate pain, obvious pain, intolerable, required to take analgesics, and sleep disturbed. Grade 3: severe pain, severe and intolerable pain, requiring analgesics, severely disturbed sleep, and may be accompanied by autonomic nerve dysfunction, showing passive posture.

### 2.4. Data Collection

Data will be collected from the anesthesia information system. Data to be collected includes patient demographics (ASA classification, age, height, weight, and gender), procedural data (type of surgery performed, length of surgery, length of anesthesia, and length of stay in PACU), and patient outcomes (any complications and adverse events in PACU). Data on the time of hospital admission and discharge were obtained from the hospital information system (HIS). The conditions of the patients, the decisions made by doctors and nurses, and the issues that needed to be or not to be addressed can be found in the PACU-related documents.

### 2.5. Data Analysis

The data were input into Microsoft Excel®2010 and analyzed after being imported into SPSS Windows (SPSS 26.0, Chicago, Illinois). The continuous variable values were expressed as mean ± standard deviation (*x* ± *s*) and compared with a 2-sample *t* test. The dichotomous data were expressed in frequency and percentage and were compared using *χ*^2^ test. If the *P* value for a two-tailed test is less than 0.05 (*P* < 0.05), it is a statistically significant result.

## 3. Results

### 3.1. Subjects' Characteristics and Baseline Equilibrium

A total of 513 patients met the eligibility criteria, including 222 patients in the pre-PACB group and 291 patients in the post-PACB group. There were no statistically significant differences between the two groups in terms of mean age, sex distribution, cardiopulmonary lesion, ASA score, tumor site, operation style, anesthesia time, operative time, and score before surgery. However, BMI in the post-PACB group was statistically significantly higher than in the pre-PACB group (*P* < 0.05) (Table 2).

### 3.2. Outcomes of Patients

The duration of intubation in the pre-PACB group was 37.7 ± 24.4 min, shorter than in the post-PACB group (42.1 ± 23.3 min, *P* < 0.05); the length of PACU stay in the pre-PACB group was 81.6 ± 31.1 min, shorter than in the post-PACB group (89.9 ± 33.5 min, *P* < 0.01); the delayed PACU stay event rate significantly decreased from (15.3%) to (9.3%) in the pre-PACB group and the post-PACB group, respectively (*P* < 0.05). But the postoperative duration of hospital stay did not significantly change over time (8.0 ± 5.8 and 8.8 ± 6.2, *P* > 0.05). Adverse events in the pre-PACB group were fewer than the post-PACB group (34.0% and 72.1%, *P* < 0.01). Although the rate of patients being unexpectedly transferred to ICU in the pre-PACB group was lower than that in the post-PACB group (1.0% and 3.2%, respectively), there was no significant difference between the two groups (*P* > 0.05) (Table 3).

### 3.3. Analysis of Adverse Events

Of the 513 subjects, 259 experienced adverse events after surgery. Severe pain (7.9% vs. 21.6%, *P* < 0.01), hypothermy (7.6% vs. 14.0%, *P* < 0.05), agitation (5.8% vs. 16.2%, *P* < 0.01), and respiratory complications (6.2% vs. 9.9%, *P* < 0.05) were the main adverse events with significant difference between the two groups. But the incidence of cardiovascular complications and nausea and vomiting was not significantly different between the two groups (*P* > 0.05) (Table 4).

## 4. Discussion

It has been reported that the quality of recovery from anesthesia can be improved by optimizing the extubation process [16], improving respiratory and circulatory conditions [17], alleviating pain [18], and managing hypothermia [19]. According to the characteristics of the elderly patients with colorectal cancer, we developed a procedure-based PACU management program using the care bundles. Besides, guided by this program, we closely followed their conditions and provided recovery care, which was proved to be effective. Compared with the patients who received conventional care, the duration of intubation and the length of stay in PACU were significantly shortened after the implementation of the program, and more adverse events such as respiratory tract, cardiovascular complications, postoperative pain, and agitation were discovered during recovery.

When the elderly patients with colorectal cancer are extubated at the early stage of recovery from anesthesia, respiratory complications, like hypersomnia, glossocoma, insufficient ventilation, respiratory depression, impaired airway protective reflex, cough with sputum, weakness, and atelectasis, are likely to occur due to delayed and residual effects of neuromuscular-blocking drug caused by the residues of anesthesia drugs and analgesics [20]. In addition, the lung inspiratory reserve capacity of elderly patients decreases significantly, which is likely to cause hypoxemia and hypercapnia. In the design of the care bundles, we incorporated the timing of extubation since admission into PACU, and attempted to improve their respiratory function before they regain consciousness to prevent atelectasis and regurgitation by elevating the head of the bed (30 degrees); low tidal volume + PEEP ventilation; according to the lung auscultation and oxygenation, we get rid of respiratory tract secretion and gave symptomatic treatment. After extubation, the patients' position was adjusted to allow for the most effective ventilation. Semi-Fowler's position (30-45 degrees) was usually recommended, with pillow cushions under patients' heads, and they were encouraged to cough and breathe deeply.

Pain assessment of elderly patients with colorectal cancer is an integral part of medical care under this management program. Individualized pain assessment should be performed immediately after patients are admitted to PACU. Early pain intervention can greatly reduce the occurrence of moderate and severe pain and postoperative agitation after extubation. Also, the effective analgesia helps the deep breath and the cough of patients and reduces the occurrence of pulmonary complications. An effective pain assessment is the first step in improving pain management. Before nurses in PACU perform pain assessment, they should be aware that anesthesia method, the use of sedatives and analgesics, and unfamiliar environments can affect the cognitive ability of patients, in addition to letting patients know about the details of the assessment before surgery. So, it is necessary to select a proper pain assessment method to relieve their pain effectively. Besides, patients should be warned of breakthrough pain, especially in the beginning of regaining consciousness.

Elderly patients with colorectal cancer have a high risk of perioperative hypothermia due to over 2 hours of operative time under anesthesia and intravenous infusion of crystalloid fluid of more than 1500 mL [21]. Hypothermia impairs coagulation function, causes more bleeding after surgery, and delays recovery from general anesthesia through pharmacodynamic and pharmacokinetic mechanisms [22]. After the implementation of this management program, we built the temperature management of the elderly patients with colorectal cancer in the operation room into our program, including the measurement of the temperature immediately after they being sent to the operation room, the monitoring of the temperature during the perianesthesia period, PACU environmental temperature setting (not less than 23°C), passive warming (e.g., cotton blanket, sheet, and insulation blanket), and active warming (e.g., pressure air-warm blanket/heater and heating of inhaled gas). After that, the occurrence of hypothermia in patients in PACU decreased significantly. The nurses took the temperature of patients during resuscitation and were aware of the risk of hypothermia. Active warming measures were immediately adopted if patients experienced chills or had bristling hair or ear temperature less than 36.0°C. Passive warming measures such as using a cotton blanket were adopted for patients with normal body temperature. If patients could communicate, they were asked if they felt fine or cold. Patients shivering from hypothermia were treated with pethidine, tramadol, or dexmedetomidine in addition to active rewarming.

The management programming of the care bundles involves many systems and people, so it is very important to manage the implementation process well. To this end, a quality management team needs to be built to ensure the program is implemented by following the steps and following the results. Besides, a complete and recognized feedback and evaluation system should be created by monitoring the movement of the patients out of bed, time of feeding, length of stay in the hospital, unexpected being transferred to ICU, and postoperative mortality.

## 5. Limitations

There are several limitations to this study. First, results from this study are retrospective and observational in nature; we are unable to identify a true causal effect of PACB on clinical outcomes. We acknowledge that during the time period of this study, some advances have been made in PACU, including increase of equipment and employees. These developments would have led to decreased length of PACU stay, thus potentially confounding our results. In addition, it is uncommon to extubate in PACU like our hospital, since extubation is often done in OR. The difference in anesthesia management may limit the external validity of the results.

## 6. Conclusion

The findings in the current study demonstrate a substantial shorten in PACU stay, along with higher event rates after implementing a PACB program. The care we describe as the PACB was the most common morbidity in PACU. The findings support our hypothesis that enhanced patients' recovery through a PACB program. They also provide additional guidance in support of PACB for elderly patients with colorectal cancer.

## 7. Relevance for Clinical Practice

In China, elderly patients with colorectal cancer undergo radical surgery increasingly, and targeted measures are needed to ensure that these patients recover well after anesthesia. The care in PACU under this program will incorporate many measures targeting the characteristics of the elderly patients into one bundle, which can provide procedure-based medical care. These measures can shorten the recovery time and improve the recovery quality after surgery. This could make the health care system more efficient, reduce unnecessary medical costs, and improve the operation efficiency of medical institutions.

## Figures and Tables

**Table 1:** Care bundles in PACU for elderly patients with colorectal cancer.

Item	Objective
Extubation procedure (post-PACB)	(1) RASS score > 2 or has regained preoperative consciousness level (2) The effect of muscle relaxants is completely reversed (3) No secretions in the airway need to be get rid of (4) Head of bed elevation by ≥30° (5) oxygenation index ≥ 150 mmHg (6) EtCO_2_ or PaCO_2_ 35~45 mmHg (7) Spontaneous breath, respiratory rate (RR) from 10~25 bpm and tidal volume 6-12 mL/kg
Circulation (post-PACB)	(1) HR < 100 bpm (2) No new onset arrhythmia (3) failing to maintain mean blood pressure >65 mmHg
Pain (post-PACB)	CPOT ≤ 4 or NRS ≤ 3
Body temperature (post-PACB)	(1) Ear temperature > 36.0°C (2) No chills, bristling hair, or coldness at the extremities (fingers, toes)
Internal environment (post-PACB)	(1) No electrolyte imbalance (2) pH 7.35-7.45 (3) No abnormal blood glucose level occurs (4) Hb ≥ 90 g/L
Pre-PACB	(1) Conventional recovery caring methods (2) Assist control ventilation and synchronized intermittent mandatory ventilation (3) ECG monitoring (4) Symptomatic treatment (5) Body temperature measurement (6) Tracheal catheter was removed after muscle strength was restored

RASS: Richmond Agitation and Sedation Scale; PACU: postanesthesia care unit; CPOT: critical-care pain observation tool; NRS: numerical rating score; bpm: beat per minute; BP: blood pressure. Yes, no, treatment.

**Table 2:** General information of patients.

	Pre-PACB group (*n* = 222)	Post-PACB group (*n* = 291)	*P* value
Gender			0.360
Male	186 (63.9%)	133 (59.9%)	
Female	105 (36.1%)	89 (39.1%)	
Age (y)	72.7 ± 5.7	73.3 ± 6.4	0.267
BMI	23.3 ± 3.3	22.6 ± 3.1	0.015
Chronic cardiopulmonary disease†	69 (23.7%)	58 (26.1%)	0.537
ASA classification			0.623
I	0	0	
II	257 (88.3%)	194 (87.4%)	
III-IV	34 (11.7%)	28 (12.6%)	
Type of operation			0.857
Radical resection for rectal cancer	119 (40.9%)	93 (41.9%)	
Radical resection for colon cancer	172 (59.1%)	129 (58.1%)	
Duration of anesthesia (min)	233.4 ± 58.6	229.8 ± 60.6	0.493
Operative time (min)	198.5 ± 58.8	194.7 ± 58.7	0.471
Score after entering PACU	4.24 ± 0.94	4.13 ± 0.70	0.119

^†^Chronic cardiopulmonary diseases: hypertension, heart disease, heart failure, asthma, chronic obstructive pulmonary disease, etc. BMI: body mass index; ASA: The American Society of Anesthesiologists; PACU: postanesthesia care unit.

**Table 3:** Outcome of patients.

	Pre-PACB group (*n* = 222)	Post-PACB group (*n* = 291)	*P* value
Intubation time in PACU (min)	42.1 ± 23.3	37.7 ± 24.4	0.040
Length of stay in PACU (min)	89.9 ± 33.5	81.6 ± 31.1	0.004
Number of patients stay in PACU over 2 h	*34* (15.3%)	*27* (9.3%)	0.040
Adverse events(cases)	99 (34.0%)	160 (72.1%)	≤0.001
Number of patients being transferred to ICU unexpectedly	*3* (1.0%)	*7* (3.2%)	0.110
Length of stay in hospital (day)	8.0 ± 5.8	8.8 ± 6.2	0.107

PACU: postanesthesia care unit.

**Table 4:** Distribution of adverse events.

	Pre-PACB group (*n* = 222)	Post-PACB group (*n* = 291)	*P* value
Respiratory complications	18 (6.2%)	26 (9.9%)	0.038
Cardiovascular complications	7 (2.4%)	9 (4.1%)	0.510
Pain	23 (7.9%)	48 (21.6%)	≤0.001
Moderate pain	18 (6.2%)	32 (14.4%)	
Severe pain	5 (1.7%)	16 (7.2%)	
RASS	17 (5.8%)	36 (16.2%)	0.003
RASSI	10 (3.4%)	21 (9.5%)	
RASSII	6 (2.1%)	11 (5.0%)	
RASSIII	1 (0.3%)	4 (1.8%)	
Nausea/vomiting	12 (4.1%)	10 (4.5%)	0.282
Hypothermy (<36°C)	22 (7.6%)	31 (14.0%)	0.020

RASS: Richmond Agitation and Sedation Scale.

## Data Availability

The data used to support the findings of this study are available from the corresponding author upon request.
